# Vocational Education Platform Based on Block Chain and IoT Technology

**DOI:** 10.1155/2022/5856229

**Published:** 2022-08-28

**Authors:** Deming Li, Rui Hu, Zhuliang Lin

**Affiliations:** ^1^School of Education, Jilin International Studies University, Changchun, Jilin 130117, China; ^2^Zhejiang Normal University, Jinhua 321004, Zhejiang, China; ^3^Xingzhi College, Zhejiang Normal University, Jinhua 321004, Zhejiang, China

## Abstract

Due to the poor effect of the traditional vocational education platform, it is difficult to meet the requirements of the current Internet education platform. To solve this problem, this paper designs a vocational education platform system based on blockchain and Internet of Things (IoT) technology. First, the system access control strategy based on blockchain technology is introduced into the teaching system so as to improve the security of the teaching system. Then, in order to solve the single point of failure and efficient transmission problems of access control in the IoT environment, this paper proposes an access control strategy based on main side chain cooperation. This strategy introduces a side chain to expand the blockchain and improve the data carrying capacity of the blockchain. To meet the requirements of high-speed data transmission, this paper designs an access control model suitable for the main side chain blockchain structure. Experimental results show that compared with other algorithms, the data request speed of the system in this paper is faster, and the storage space is smaller. Therefore, the proposed technology based on blockchain and IoT can meet the use requirements of vocational education platforms.

## 1. Introduction

“Education is the foundation of the development of science and technology.” Today's world is dominated by information technology, especially the IoT ushered in the era of the Internet of everything [1]. The outbreak of COVID-19 in 2020 also indirectly promoted the boom of online education. It changes the rigid system of time and place between teachers and students and makes learning methods diversified and more humanized [2]. Since entering the 21st century, China's education industry has developed rapidly. With the high attention paid to informatization, online vocational education has gradually come into people's sight and has been gradually accepted by most people [3]. This greatly supports and further optimizes the online education industry. From a global perspective, online vocational education is gaining momentum, but there are still many problems [4]. For example, information asymmetry, difficulty in resource matching and docking, difficulty in safeguarding IP content, high transaction costs, and other phenomena still hinder the progress of online vocational education in many cases, which are several shortcomings of the industry.

Blockchain is a database that arranges data groups in a specific sequence based on time sequence [5], and it follows the techniques of cryptography to protect data security. It contains information, including historical transaction data, etc., which is an open and long-standing information block occurring in a certain established group [6]. To some extent, the core elements of blockchain technology include blockchain data structure, distributed node consensus algorithm, means of cryptography, intelligent contract composed of automated script code, distributed infrastructure, computing methods, etc. [7]. The above elements guarantee the data characteristics of blockchain technology, such as the generation, validation, storage, and updating of data, as well as the security of data [8]. At the same time, blockchain also has the advantage of decentralization. In today's world, the most prominent application of this technology is Bitcoin [9]. Its advantage lies in the reduction of intermediate links, and the docking of currency passwords is more convenient.

As far as the current Internet technology is concerned, there are still many problems in the development of vocational education platforms, such as information asymmetry, unrecognized educational experience, certificates, etc. With the development and gradual maturity of blockchain technology, it has emerged in the field of vision of relevant industries and is involved in credit endorsement, information encryption, contract, and other aspects. There is also a high space for development in the education industry [10]. This technology is often used in the education industry: (1) Distribute learning record storage. (2) Provide an authoritative, low-cost certification system for online education. (3) Instead of smart contracts, play the role of education contracts and vouchers. (4) Store educational resources and scientific research achievements instead of certificates such as copyright certificates. (5) As knowledge currency, play the role of the decentralized world knowledge base.

The industrial information revolution and the development of the Internet have revolutionized the education model. Learning methods, such as distance education and online courses, have mushroomed. As the proof of virtual assets, blockchain undertakes the process of knowledge asset circulation among teachers, students, and even families [11]. However, the education blockchain forms the proof of knowledge asset circulation, storing all kinds of data in the online education community. The personnel composition of the educational blockchain includes providers, learners, and propagandists [12]. Data storage can be used to record the activity of the various parties in the community, which in turn encourages them to be more proactive, making the community and the education system work well and benefit from it all.

The rise of blockchain technology has aroused widespread interest in academia, politics, and business. Various advantages of this technology will certainly achieve excellent results and effects in the education industry [13]. Especially in the vocational education platform, its values and approaches mainly include the following:

1. Promote the healthy, efficient, and sustainable use of open education resources (OER). The education industry in the 21st century is changing with each passing day, with abundant resources. Both teachers and students have more convenient digital resources [14]. However, problems, such as copyright awareness and miscellaneous resources, are also plaguing people. How to create a healthy, efficient, and sustainable education resource system is the difficulty and pain point in the field of OER in the real world. Blockchain technology can effectively solve problems; thus, OER has the opportunity to move to new heights.
2. To form a student information database and build a new mechanism of education and learning. The memory ability of blockchain technology can completely record students' information and keep it as an archive for life [15]. Educational organizations can record or retrieve relevant personnel data in the database without space and system constraints, which greatly reduces the phenomenon of imperfect credit and school-society disconnection in the education industry.
3. Build a decentralized education platform to promote educational equity. At present, most of China's education industry is public education; education resources are controlled by the government and public schools. However, people's knowledge level or learning status of a certain subject must be verified by relevant academic qualifications and diplomas. But diplomas and degrees are not accurate proof of one's ability. Therefore, decentralization contributes to education equity and prevents monopoly [16].
4. Achieve the “true self-organization” operation of online education. The combination of blockchain technology and network learning is the development direction of the two industries for a period of time in the future, with a relatively bright future. Blockchain technology can improve and restructure online education networks to achieve the “true self-organization” operation of online education.

As most existing education systems adopt a centralized management approach, they face many challenges in scalability, data security and privacy, multiparty collaboration, and data sharing. Blockchain technology can fundamentally ensure the data integrity, security, and sustainability of vocational education platforms. IoT technology utilizes existing network infrastructure to integrate various physical devices with the Internet to realize information exchange between things and things and between things and people. In view of this, this paper designed a vocational education platform system based on blockchain and IoT technology.

The innovations and contributions of this paper are listed as follows:

1. The system access control strategy based on blockchain technology is introduced into the teaching system so as to improve the security of the teaching system.
2. In order to solve the single point of failure and efficient transmission problems of access control in the IoT environment, this paper proposes an access control strategy based on main side chain cooperation. This strategy introduces a side chain to expand the blockchain and improve the data carrying capacity of the blockchain.
3. In order to meet the requirements of high-speed data transmission, this paper designs an access control model suitable for the main side chain blockchain structure.

This paper consists of four main parts: the first part is the introduction, the second part is the methodology of vocational education platform based on blockchain and IoT technology, the third part is the result analysis and discussion, and the fourth part is the conclusion.

## 2. Methodology

### 2.1. Teaching System Design Based on IoT Technology

The construction of teaching modules with the help of IoT technology can change teachers' traditional teaching methods. Making full use of network technology can make teaching more colorful and solve the problem of boring course content. The module of vocational education mainly includes intelligent classrooms, intelligent equipment, intelligent courses, and so on. IoT mainly through the optimization of teaching resources improves the management of the classroom, laboratory, and other teaching resources. IoT can combine these hardware facilities with the Internet so as to achieve a new level of vocational education.  Figure 1 is the vocational education module based on IoT technology.

The IoT in the library is also one of the module construction contents of vocational education, which makes use of the IoT to manage the library digitally and make the library develop in the direction of intelligence. Even though the library has a wide range of reading resources, the location of books can be found quickly through IoT technology. This greatly improves the guiding effect of the library but also relieves the pressure on the library staff.

In the module design of this paper, vocational education is established in the IoT technology to realize the concept of “people-oriented.” It integrates teaching, logistics, life, and technology departments on campus through IoT technology. Through the vocational education platform, all kinds of information and items on campus are integrated to realize the interconnection between people, people, and things, and things and things so as to serve teachers and students.  Figure 2 shows the overall module structure of vocational education based on IoT technology in this paper.

### 2.2. System Access Control Method Based on Block Chain

In the domain of IoT, access control needs to be able to respond and reply quickly to requests. The commonly used approach in the access control strategy using blockchain in the field of IoT is to divide the architecture into two parts: the blockchain side and the IoT device side [17]. However, in the field of Educational IoT, there are not only a large number of nodes, but also many nodes do not need to complete both resource requests and upload them at the same time. At the same time, much of the educational data is of great importance to students, so it is important not only to verify the security of the access control model but also to verify the security of each device connected to the IoT.

In view of the above access control architecture problems in the field of Educational IoT, this paper designs a strategic architecture for Educational IoT, as shown in Figure 3. The architecture is based on the usage of resources in the client, blockchain network, and equipment end three parts, and the client and the device side is the resource of the uploading and requester, respectively. Among them, the client is responsible for authorization upload, strategy, and resource use of resources. At the same time, the client configuration with blockchain connects SDK and realizes the client with the blockchain network connection. The devices in this part are usually some edge terminals with weak computing capabilities. Therefore, they are connected with the blockchain network through the gateway to send requests for resources. By unifying the request flow of each terminal and separating it, the conflict of request is avoided, and the high-speed transmission of requests is realized.

The blockchain network is the main logical part of the strategy. The authentication of IoT devices is designed; that is, the terminals connected to the blockchain network need to be logged in and verified in advance before they can be allowed to connect. By analyzing the data confirmation process of Ethereum, it can be found that every operation on Ethereum requires a full node confirmation, which is the main reason for the low throughput of Ethereum. However, in the environment of Educational IoT, due to the batch of repeated requests of terminal operation, it does not need to confirm the whole node for each operation but only confirm the key operations. Therefore, in this paper, the blockchain puts the smart contract module on the side chain, and the side chain executes the access control strategy. The data of the side chain is packaged and sent to the plasma contract connected to Ethereum through the miner operator and sent in batches. As the main chain, Ethereum only needs to obtain the hash value of the transaction through the plasma contract in batches and synchronize it to Ethereum for locking, which not only improves the speed of access control but also realizes decentralized access control.

In the access control of Educational IoT, we should not only have a simple and clear division of authority but also prevent the risk of overauthorization and privacy data disclosure. Therefore, it is necessary to divide access control permissions according to the characteristics of use scenarios. For the Educational IoT scenario, the most important thing is to prevent data leakage. Although researchers design some methods for common models, such as role set and permission set, to prevent illegal access, this method has high requirements for the design of protection measures. If the prevention method is cracked, the lawless person can quickly obtain various data resources, causing the students to suffer irreparable losses. In order to prevent data leakage more effectively, this paper designs an access control model based on master side chain cooperation. Each access request can be separated from the source of the received data so as to achieve the effect of preventing the data from being leaked.  Figure 4 is the model architecture.

In the part directly connected with the subject and object, the model designs the subject information point and object information point. The subject information point is the access control execution point interacting with the subject, which is responsible for transmitting the subject's access request and subject information, as well as returning the execution result after processing the request. The object information point is the execution point of interaction with object resources and is responsible for collecting object and resource attributes. When an access request occurs, it uploads the required object resource information for the reference of the access control strategy. This design blocks the direct access of external entities to the interior of the model and avoids illegal intrusion. At the same time, the output of data is directly returned to their connected entities through the execution point, which effectively avoids the leakage of data because the design of the information processing point is to separate the execution and storage of access control policy. When a request occurs, the processing point directly calls the designed access control policy to judge the request. The processing point only has permission to call the access control policy and cannot modify the policy. The permission to view the policy every time will be withdrawn after completing this access request, which effectively avoids the disclosure of the access control policy.

This paper completes the decision-making authorization and decision-making information management of access control authority through three smart contracts deployed on the side chain. The three contracts are precontract, access control contract, and supervision contract, respectively. The interaction mode of the contract is shown in Figure 5.

On the side chain, the head of the blockchain deploys the precontract, which maintains a table of information about regulatory and access control contracts. A monitoring contract is then deployed on the next block, which contains a time-tolerance function to monitor the frequency of visitors and allows bulk access to a specified range of access. At the same time, the monitoring contract maintains a list of offending visitors that can be recorded and disciplined. After the block is used for access control contracts, each blockchain connects different Internet equipment, access control, contract maintenance access strategy table, and access records; when there is an access request, access control can access strategy as defined by the contract, and the test results of regulatory contracts, responding to the access request, and when there is a new access control policy to join, keep adding new access control contracts to the chain.

To prevent data from being tampered with, the blockchain requires simultaneous validation of the data. The algorithm in [18] is used in blockchain. In this algorithm, the hash value of each data is calculated through the hash algorithm, and only the root hash generated in the blockchain can be synchronized to verify the data. However, this algorithm also has disadvantages. It can be very difficult to verify that certain data does not exist in the block. Therefore, the Plasma Cash framework uses the algorithm in reference [19], which arranges the data on the chain according to the sequence of element numbers to form an ordered sequence of leaf nodes. When there is no transaction somewhere, the leaf node stores a null value directly. When you need to verify the nonexistence of data, you only need to search the data location and find the empty location to complete the nonexistence proof. After the access control information is stored on the side chain, hash locking is performed using the algorithm in Literature [19], and the Markel root is synchronized to the Ethereum main chain. Once the information is tampered with, Merkel root will also change. The main chain is responsible for data verification, while the side chain is responsible for data storage and request processing, which not only ensures the authenticity of the data but also greatly improves the throughput rate of the blockchain. The algorithm flow of literature[19] is shown in Figure 6.

In the Ethereum blockchain, attackers attacking the consensus mechanism to modify the block data is the main reason why the security of the blockchain is threatened. This paper adopts the attack model proposed in [20] to analyze the security of the Ethereum blockchain by taking the POW consensus mechanism commonly used by researchers as a use case. The stochastic binomial process is used to describe the competition between the trust chain and attack chain faced by the Ethereum blockchain. The attacker offsets the *k* block gap by making the forgery chain longer than the trust chain. Among them, the probability of successfully offsetting the *k* block gap is similar to Gambler's Ruin Problem (GRP). The probability that the length of the attack chain at the time of the successful attack is not less than the length of the trust chain. The calculation is as follows:

(1) $$\begin{array}{c} v_{k}=\left\{\begin{array}{cc} 1\text{,} & u\leq v\text{,}\\ {\left(\frac{v}{u}\right)}^{k}\text{,} & u>v\text{,} \end{array}\right. \end{array}$$

where *u* is the probability that the trusting node gets the next block accounting right, *v* is the probability that the attacking node gets the next block accounting right, *u*+*v*=1.

To obtain the exact number of block progress of the attack chain, the potential progress of the attack chain can be regarded as a Poisson distribution, assuming that it will take the average expected time for the trust chain to produce a block. The expected value of the distribution is expressed in (2) as follows:

(2) $$\begin{array}{c} \lambda =k\cdot \frac{v}{u}\text{.} \end{array}$$

In order to calculate the probability that the attack chain length reaches the trust chain length, the Poisson distribution probability density of the progress number of attack chain blocks is multiplied by the probability that the attack chain length still reaches the trust chain length under this number. The probability *u* of the attacker successfully tampering with block data is represented by the following:

(3) $$\begin{array}{c} U=\overset{\infty }{\underset{z=0}{\sum }}\frac{\lambda^{z}\cdot e^{-\lambda }}{z!}\cdot \left\{\begin{array}{cc} {\left(\frac{v}{u}\right)}^{\left(k-z\right)}, & z\leq k,\\ 1, & z>k. \end{array}\right. \end{array}$$

In order to avoid infinite summation of (3), it is further transformed into the following:

(4) $$\begin{array}{c} U=1-\overset{k}{\underset{z=0}{\sum }}\frac{\lambda^{z}\cdot e^{-\lambda }}{z!}\cdot \left(1-{\left(\frac{v}{u}\right)}^{\left(k-z\right)}\right)\text{.} \end{array}$$

## 3. Result Analysis and Discussion

In order to verify the feasibility of the proposed algorithm, a test cloud computing environment was set up in the laboratory. In the cloud environment, a server cluster consists of five workstations with Intel Corei7 CPUs, 128 GB DDR4 memory, 512 GB, and SSD disks. Docker running environment is deployed on the cluster, and data sharing system is run based on hyperledger fabric blockchain platform. Statistics of various indicators of system operation, all data is the average of 10 experiments.

The simulation system simulates users uploading files to the cloud and authorizes file access rights to the data requester via blockchain. There are two servers running: public chain service and private chain service, respectively. There are 100 simulated data requesters.  Figure 7 shows the time curve required by data request nodes on the public chain from request to data acquisition. As the number of requesting nodes increases, the data synchronization time of nodes is roughly stable. It shows that the system proposed in this paper is more effective for file sharing.

In terms of block generation efficiency, the total number of blocks increases, see Figure 8. According to the simulation data, the generation time of a single block shows an upward trend, which is because the consensus algorithm in the blockchain needs to be synchronized among the members of the whole chain. As the algorithm in this paper adopts a secure data sharing model and algorithm, the average generation time is within a controllable range.

Table 1 compares the algorithm of this paper with several research results from five perspectives, and it can be seen that this model has certain advantages on the whole.

With the increasing number of devices and requests in the Educational IoT, the code volume of access control contracts is also increasing rapidly, putting great pressure on the storage of blockchain. The size and growth rate of storage space usage vary depending on the architecture of access control policies. Therefore, the storage stress on the blockchain should be fully considered when designing the access control contract. Currently, the commonly used prevention and control strategies mainly include literature [22] and literature [23]. Literature [22] associates roles with permissions and users obtain corresponding permissions through roles given by the system. It can support cross-domain control and device heterogeneity in the IoT environment. The strategy in literature [23] takes attributes as the key element to control permissions and implements dynamic node secure access through attribute association permissions. In order to analyze the storage pressure caused by the access control strategy on the blockchain, two commonly used access control strategies are designed and compared with the proposed strategy to analyze the increase of the contract size with the number of devices. The contract information is shown in Table 2.

Assume that the number of devices is *t,* and each device initiates access control requests. In this case, for every *g* contract deployed on the device in the access control policy, *g* host and object pairs are generated. That is, *t*^*g*^ contracts are deployed in this policy. From this, we can get the expression that the contract size increases with the number of devices.

The strategy formula of this paper is as follows:

(5) $$\begin{array}{c} f\left(i\right)=65.13i+65.05\text{.} \end{array}$$

The strategy formula in literature [22] is as follows:

(6) $$\begin{array}{c} a\left(i\right)=20.5i^{2}+34.9\text{.} \end{array}$$

The strategy formula in literature [22] is as follows:

(7) $$\begin{array}{c} b\left(i\right)=180.13i+160.07\text{.} \end{array}$$

Draw the function image as shown in Figure 9 according to the function expression. As can be seen from Figure 9, the code quantity of the strategy in literature [22] increases rapidly with the increase of the number of devices, and it is higher than the strategy designed in this paper if the number of devices is above 4. Although the code growth rate of the strategy in literature [23] is lower than that of the strategy in [22], the growth rate is still fast compared with the strategy in this paper. Compared with other common strategies, the strategy proposed in this paper not only ensures data transmission efficiency but also saves a lot of storage space, which is more suitable for the application scenarios of massive nodes of the Industrial IoT.

The generation time of access control policy is an important index to measure the quality of the access control model. To verify the effect of the proposed model in policy generation, a traditional blockchain IoT access control model is designed to conduct a comparative experiment. Test the model in this paper and several other models, and record the average time for this number of visits. As the side chain does not require block confirmation, in order to more intuitively see the generation speed of the model control strategy, the model in this paper is put on the Ethereum test chain for the experiment (see Figure 10).

The generation time of the policy has a high rise with the increase of the number of concurrencies. However, the main side chain cooperative access control model proposed in this paper can generate access policies more quickly, and the delay of policy generation tends to be stable at high-frequency access. According to the experimental data, the model in this paper is more suitable for the application of massive terminal nodes of the Educational IoT.

In this paper, Matlab 2018b is used for simulation, and the experimental results are shown in Figure 11. From Figure 11, it can be seen that the probability of success of the attacker tampering with block data decreases with the increase of block difference *k*. When the number of blocks difference is the same, the probability of the attacker's success in tampering with block data increases with the probability of obtaining the accounting right of the next block (that is, the computing power). Therefore, when the attacker has more arithmetic power, it is more likely to tamper with the block data and turn itself into a chain of trust. Therefore, the effectiveness of the attacker's attack can be reduced by increasing the number of trust chain blocks so that they are long enough and by increasing the arithmetic power. Due to a large number of devices typically present in an IoT ecosystem, each device can act as a light node in an Ethereum blockchain with Turing-complete properties. Therefore, the IoT device access control mechanism based on the Ethereum blockchain in this paper meets the security requirements of the IoT ecosystem for device access control.

## 4. Conclusion

The traditional vocational education platform has some problems, such as insecure data, low credibility, asymmetric information, and difficult resource matching and docking. In response to the above issues, this paper designs a vocational education platform system based on blockchain and IoT technology. Firstly, the system access control strategy based on blockchain technology is introduced into the teaching system in this paper so as to improve the security of the teaching system. Then, an access control strategy based on main side chain cooperation is proposed to solve the single point of failure and efficient transmission problems of access control in the IoT environment. Finally, in order to meet the requirements of high-speed data transmission, this paper designs an access control model suitable for the main side chain blockchain structure. The experiment proves that the technology based on blockchain and IoT proposed in this paper can effectively realize the credible and efficient operation of practical teaching activities on vocational education platforms. However, at present, blockchain technology is still not mature, the infrastructure is not perfect, and the cost of information transmission is still relatively high. In order to achieve real implementation and support the relevant business in the field of education, there will be many technical implementation problems that need more in-depth research and exploration.

## Figures and Tables

**Figure 1:** Vocational education teaching module based on IoT technology.

**Figure 2:** Overall architecture of vocational education platform construction module.

**Figure 3:** Strategic architecture of Educational IoT.

**Figure 4:** Architecture of access control model.

**Figure 5:** Interaction way of contracts on the sidechain.

**Figure 6:** The algorithm flow.

**Figure 7:** Data request node access performance curve.

**Figure 8:** Block generation efficiency diagram.

**Figure 9:** Comparison of access control contract storage space growth.

**Figure 10:** Comparison of generation speed of four models.

**Figure 11:** Comparison algorithm of attack success probability.

**Table 1:** Comparative analysis of algorithms.

Algorithms	Based on the blockchain	Consensus mechanism	Reduce the stress on the main chain	Private chain	Block generation efficiency
Literature [21]	No	—	Yes	No	Good
Literature [22]	Yes	POW	No	No	Low
Literature [23]	Yes	POI	No	Yes	Medium
Proposed	Yes	DPOS	Yes	Yes	Optimal

**Table 2:** Related information of smart contract.

Strategies	Other contracts		Equipment contract		Total contract code
	Contract	Contract size	Contract	Contract size	
Proposed	Precontract	38.36			130.18
	Regulatory contract	26.52			
	Access control contract	65.3			

Literature [22]	Related contract 1	12.4	Access control contract		55.40
	Related contract 2	9.6		20.50	
	Related contract 3	12.90			

Literature [23]	Related contract A	80.50			340.20
	Related contract B	42.8			
	Related contract C	36.77			
	Access control contract	180.13			

## Data Availability

The labeled dataset used to support the findings of this study is available from the corresponding author upon request.
